# Impairment of Lung Function Increases the Risk of Postoperative Respiratory Failure for Esophageal Carcinoma: A Systematic Review and Meta-Analysis

**DOI:** 10.1155/2021/5327682

**Published:** 2021-11-30

**Authors:** Yanming Sun, Ying Zhu

**Affiliations:** Department of Intensive Care Unit, Affiliated Hangzhou First People's Hospital, Zhejiang University School of Medicine, Hangzhou, Zhejiang, China

## Abstract

**Objective:**

To study lung function impairment by meta-analysis to increase the risk of postoperative respiratory failure in patients with esophageal carcinoma.

**Methods:**

We searched PubMed, ScienceDirect, and CNKI and other databases, and the search time was set to the time the database was established. We screened the relevant literature to study the relationship between lung function damage and postoperative respiratory failure in patients with esophageal cancer, determined to include the literature and extracted relevant data, and then, applied NOS. The scale evaluates the quality of the literature, and the ReviewManager software was used to perform meta-analysis on the extracted data.

**Results:**

Finally, 9 related articles and 2822 research subjects were included, and the average score of literature quality was 5.78 points, the heterogeneity of the literature was large (*I*^2^ = 84%), the random effects model was used for analysis, and the correlation between the two showed SMD = 0.09, 95%CI[−0.09, 0.31], *Z* = 1.10, *P* = 0.27, which is consistent with the results of the subgroup analysis.

**Conclusion:**

The results of the study show that lung function impairment has a positive relationship with postoperative respiratory failure in patients with esophageal cancer. Pulmonary function impairment in cases with different case characteristics can also aggravate the severity of respiratory failure.

## 1. Introduction

According to relevant statistics, about 300,000 people die from esophageal cancer each year, which has become a gastrointestinal malignant tumor with a high incidence rate in the world, and China is a typical high-incidence area [1]. Patients with early- and middle-stage esophageal cancer usually choose surgery as the preferred treatment. Surgery can completely remove cancer lesions and clean lymph nodes, so as to inhibit the spread of cancer cells and realize the rehabilitation of patients [2]. Surgery for esophageal cancer is very traumatic, and its complications such as respiratory failure are prone to occur after surgery. This is also one of the main reasons for postoperative death of patients. Foreign scholars [3] reported that the incidence of respiratory failure after esophageal cancer surgery was 33%–38%, and domestic reports were 14.6%–30.8% [4, 5]. In recent years, a number of studies have analyzed the risk factors of postoperative respiratory failure for esophageal cancer. The results mainly include patient age, BMI, smoking index, operation time, lung function damage, and postoperative complications. However, some conclusions, especially lung function damage, are still controversial in the academic community. For this reason, this study conducted the following systematic analysis on the risk of lung function damage after esophageal cancer postoperative respiratory failure.

## 2. Materials and Methods

### 2.1. Meta-Analysis Steps

1. The problem that the meta-analysis wants to solve is concisely and clearly put forward
2. According to the purpose of this meta-analysis, the criteria for inclusion and exclusion of the literature are determined
3. Appropriate search strategies are developed to collect relevant research
4. The retrieved documents are deduplicated and screened
5. The NOS scale is used to evaluate the literature quality of the selected literature
6. Relevant data are extracted from the included literature according to the premade tables
7. Review Manager and other statistical software are used to perform statistical analysis on the data extracted from the included literature
8. The result is obtained through statistical analysis, and the result is explained in detail
9. The database is searched again in the same way to maintain and update the literature

### 2.2. Search Strategy

The search databases are PubMed, Science Direct, and CNKI. Chinese search terms include esophageal cancer, postoperative respiratory failure, and lung function damage; English search terms include esophageal cancer, postoperative respiratory failure, lung function damage, postoperative esophageal cancer, and esophageal cancer. Complications are searched by “OR” and “AND.” See Table 1 for subsequent specific search strategies.

### 2.3. Inclusion and Exclusion Criteria

#### 2.3.1. Inclusion Criteria

(1) The English literature published since the establishment of the literature database; (2) the main confounding factors were controlled in the research; (3) the research design was reasonable; (4) there was clear information on lung function damage; and (5) patients with respiratory failure after esophageal cancer confirmed pathologically [6–8].

#### 2.3.2. Exclusion Criteria

(1) Articles in languages other than English; (2) documents with repeated reports; (3) articles with poor research design and substandard quality; (4) studies with incomplete data required; (5) reviews and systematic evaluative literature; (6) literature with few subjects included; and (7) studies without a control group [9–11].

### 2.4. Selection of Articles for This Systematic Review and Extraction of Data

#### 2.4.1. Selection of Studies for This Systematic Review

1. We import the documents retrieved from the database according to the preestablished search strategy into the EndNote software for deduplication.
2. We read the titles and abstracts of the remaining documents after deduplication and preliminarily screened out documents that do not meet the inclusion criteria according to the established inclusion and exclusion criteria, such as documents that are not related to the subject, documents with non-human subjects, and languages other than Chinese and English Literature.
3. We download the full text of the remaining documents and quickly read and exclude unnecessary documents, such as documents with incomplete data and documents with only cases in the research object. The remaining documents after this step are included in the meta-analysis [12].

#### 2.4.2. Extraction of Data

After carefully reading the full text of the included literature, we extracted the data according to the predesigned table. The data extracted from the included literature in this article include basic information of the included literature (first author and publication year) and research information of the included literature (research area, case group/control group, and randomized controlled experiment method). Finally, we recorded the extracted data in a predesigned form [13].

### 2.5. Assessment of Quality

We carefully read the full text of the included literature. The included literature in this article is a case-control study. The Newcastle–Ottawa Scale (NOS) can be used to evaluate the quality of the included literature. The NOS scale consists of three parts and 8 questions. The full score for the evaluation of the quality of the literature is 9 points. When the literature score is 5 points or more, it means that the quality of the literature is good; when the literature score is less than 5 points, it means that the document is of good quality. If the quality of the literature is poor, it can be excluded in the literature screening [14].

### 2.6. Statistical Analysis

#### 2.6.1. Choice of Effect Model

The choice of random-effects model or fixed-effects model is determined based on *I*^2^. First, we import the data extracted from the included literature into the Review Manager software and select the random-effects model to make a forest plot to obtain *I*^2^. *I*^2^ is an important value to measure the degree of heterogeneity between studies. The larger the *I*^2^, the greater the heterogeneity between the studies. On the contrary, the smaller the *I*^2^, the smaller the heterogeneity between the studies. When *I*^2^ ≤ 50% (*P* ≥ 0.1), it means that the heterogeneity between the studies is small, and the fixed-effects model is used for meta-analysis; when *I*^2^ > 50% (*P* < 0.1), it means the heterogeneity between the studies. It is highly sexual, and the random-effects model is used for meta-analysis at this time.

In addition, due to the different measurement units included in this meta-analysis, the standardized mean difference SMD was selected when the effect size index was selected.

#### 2.6.2. Treatment of Heterogeneity (Subgroup Analysis)

Subgroup analysis is to divide the included literature into multiple subgroups for analysis based on multiple characteristics. For example, we divide the included research into multiple subgroups according to the age of each research object and see whether the results of each subgroup change, to properly explain the impact of age on the final results, or divide the included literature into different subgroups according to their scores, to see whether the quality of the literature has an impact on heterogeneity. The nine articles included in this study were divided into multiple subgroups based on the following characteristics to conduct subgroup analysis to find the source of heterogeneity:

1. According to the research race, they are classified into Asians and Europeans and Americans
2. Classification according to the number of cases included in the study
3. Classification according to the quality of the literature

#### 2.6.3. Heterogeneity Treatment (Sensitivity Analysis)

Sensitivity analysis means that according to the characteristics or types of each study included in the meta-analysis, by excluding certain studies, the impact on the meta-analysis is explored. Sensitivity analysis can eliminate the included documents one by one and explore whether each document has a significant impact on the results. If a document is eliminated, the results of the literature have changed significantly, and the reasons for the significant impact of the literature on the overall results can be further analyzed.

## 3. Results

### 3.1. Literature Screening Results

1. In April 2021, a document search was conducted in PubMed, ScienceDirect, and CNKI based on a preestablished search strategy, and 163 documents were obtained after preliminary search.
2. We imported the obtained documents into EndnoteX9 software to remove 24 articles, and finally, 139 articles remained.
3. According to the inclusion and exclusion criteria, we preliminarily read the title and abstract of the literature, eliminated 108 articles, and finally, left 31.
4. Finally, we carefully read the full text of the literature, eliminated the literature with incomplete data, and finally, included 9 articles. The specific screening process is shown in Figure 1.

### 3.2. Data Extraction and Quality Evaluation

This article included a total of 9 studies, including three studies from China, three studies from the United States, one study from Denmark, one study from Japan, and one study from Mexico. A total of 2822 people were enrolled in 9 studies, including 1436 patients with lung function impairment and 1386 controls. According to the NOS scale, the quality of the included literature was scored, and the average score of the included literature was about 5.78 (Table 2).

### 3.3. Meta-Analysis Results

#### 3.3.1. The Relationship between Lung Function Damage and the Risk of Respiratory Failure after Esophageal Cancer Surgery

A total of 9 articles were included in this meta-analysis, with a total of 2822 research subjects. The final results showed that lung function damage has a certain effect on respiratory failure of patients after esophageal cancer surgery (SMD = 0.09, 95% CI (−0.09, 0.31), *Z* = 1.10, *P* = 0.27), and the result is shown in Figure 2. The research heterogeneity is high (*I*^2^ = 84%), so subgroup analysis or sensitivity analysis is needed to find the source of heterogeneity.

#### 3.3.2. Results of Subgroup Analysis

Due to the large heterogeneity of this meta-analysis, subgroup analysis is needed to find the source of heterogeneity. The included literature was divided into several groups for subgroup analysis according to study race, number of included cases, literature quality, and so on. The specific results are summarized as follows:

1. Subgroup analysis is performed according to different research races. According to *I*^2^ = 84%, a random-effects model is selected for analysis. The results showed that this heterogeneity mainly comes from research conducted in Asia (Asians, *I*^2^ = 93%; Europeans and Americans, *I*^2^ = 43%). The heterogeneity of the studies conducted in Europe and America is relatively low, and the results of the two groups are statistically significant, as shown in Figure 3.
2. Subgroup analysis is performed according to the number of cases included in different research cases. According to *I*^2^ = 84%, a random-effects model is selected for analysis. The results showed that this heterogeneity mainly comes from studies with more cases. The heterogeneity of studies with fewer cases included is relatively low, and the results of the two groups are statistically significant, as shown in Figure 4.
3. Subgroup analysis is performed according to different research qualities. According to *I*^2^ = 84%, a random-effects model is selected for analysis. The results show that this heterogeneity mainly comes from lower-quality research (lower-quality research *I*^2^ = 95%; higher-quality research *I*^2^ = 33%). The high-quality studies have relatively low heterogeneity, and the results of the two groups are statistically significant, as shown in Figure 5.

### 3.4. Sensitivity Analysis Results

The random-effects model was used for sensitivity analysis after the included studies were eliminated one by one. The specific results are shown in Figure 6. It can be seen from the figure that when the literature whose first author is Wenlong Huang is excluded, the overall heterogeneity is significantly lower (*I*^2^ = 84% becomes *I*^2^ = 47%). Therefore, the sensitivity analysis results show that the heterogeneity is mainly caused by the first author Wenlong Huang's literature. After reading the full text again, the analysis may be due to the fact that the selected case treatment methods in this study are different from those of other studies.

## 4. Discussion

Esophageal carcinoma is a common cancer [10]. Surgery is the first choice for treatment [13]. However, surgical treatment could be harmful to the patient's body organs and result in a series of complications until death [14]. Among them, respiratory failure is one of the most serious complications after surgical treatment, and the incidence rate is as high as 30% according to survey [15, 16]. Though respiratory failure is difficult to predict and control, if it cannot be effectively controlled after surgical treatment, it is likely to endanger the lives of patients. Several studies have shown that lung function damage is one of the important indicators of postoperative respiratory failure in patients with esophageal cancer. Yoshida et al. [17] believed that chronic obstructive pulmonary disease (COPD) or diabetes is the main cause of postoperative respiratory failure in patients with esophageal cancer. Other scholars pointed out that preoperative pneumonia, tuberculosis, acute respiratory distress syndrome (ARDS), and other diseases in patients with esophageal cancer could make them more prone to respiratory failure [18–20]. The results of this meta-analysis initially show that esophageal cancer patients with preoperative lung function impairment are more likely to suffer from respiratory failure after surgical treatment, and lung function impairment may be a risk factor for respiratory failure.

This meta-analysis conducted a literature search in Pubmed, ScienceDirect, and CNKI based on a preestablished search strategy and finally included 9 related articles. Three studies were conducted in China, three in the USA, one in Japan, one in Mexico, and one in Denmark. The total sample size was 2822: intervention group = 1436; control group = 1386.

According to the NOS scale for literature quality scoring, the average score (5.78 points) is relatively high. The heterogeneity of this meta-analysis is very high (*I*^2^ = 84%), so a random-effects model was used to conduct a combined analysis, and subgroup analysis and sensitivity analysis were used to explore the source of heterogeneity.

This meta-analysis was divided into several subgroups according to race, number of included cases, and literature quality sources.

Although the results of each subgroup analysis are not completely consistent, all show that lung function impairment is related to the risk of respiratory failure after esophageal cancer surgery. The subgroup showed that lung function impairment has a significant impact on the risk of esophageal cancer.

This meta-analysis has several advantages: firstly, this study includes studies not only from developed countries but also from developing countries. Secondly, we excluded studies that included fewer cases (*n* < 50) to minimize the impact of small studies on the results. Thirdly, the quality of the included studies is sufficient (average = 5.78).

Although this study strictly formulated the literature retrieval strategy and inclusion and exclusion criteria and carried out a more systematic and comprehensive literature retrieval and literature screening, it also has certain limitations.

Only three databases of Pubmed, ScienceDirect, and CNKI were included. Only one author conducted retrieval, screening, and quality assessment of the literature. When the data were combined, other factors for postoperative respiratory failure for esophageal cancer were not considered. The number of documents included in this article was small (9), and the included studies had high heterogeneity, and the heterogeneity in the overall analysis and subgroup analysis was relatively high. Therefore, the literature included in this article is not enough to directly prove the research. More high-quality studies are required to further validate the results.

## Figures and Tables

**Figure 1:** Flow chart of literature screening.

**Figure 2:** Correlation between lung function impairment and risk of respiratory failure after esophageal cancer surgery.

**Figure 3:** Analysis of the correlation between lung function impairment and the risk of respiratory failure after esophageal cancer surgery in different ethnic subgroups.

**Figure 4:** A subgroup analysis of the correlation between lung function impairment and the risk of respiratory failure after esophageal cancer surgery.

**Figure 5:** Different quality subgroup analysis of the correlation between lung function impairment and respiratory failure risk after esophageal cancer surgery.

**Figure 6:** Sensitivity analysis of the correlation between lung function impairment and the risk of respiratory failure after esophageal cancer surgery.

**Table 1:** Search strategy.

Search	Add to builder	Query	Items found
#5	Add	Search (#1 AND #2) Filters: Publication date from creation date to 2021/09/01; Humans	114
#4	Add	Search (#1 AND #2) Filters: Publication date from creation date to 2021/09/01	131
#3	Add	Search (#1 AND #2)	306
#2	Add	Search (Esophageal cancer OR lung function damage)	20710
#1	Add	Search (postoperative respiratory failure OR lung function damage OR postoperative esophageal cancer OR esophageal cancer complications)	435753

**Table 2:** Features of included studies and quality assessment results.

Serial number	Included studies	Region	Case/control	Core
1	Adrianne K., 2014	USA	75/95	6
2	Carol Rubin, 2006	USA	63/63	6
3	Hiroaki Itoh, 2009	Japan	403/403	5
4	Huaizhuang Ye, 2009	Zhejiang, China	78/72	6
5	Maria Wielsoe, 2017	Greenland	77/84	6
6	Nicole M. Gatto, 2007	USA	355/327	7
7	Rogelio Recio-Vega, 2011	Mexico	70/70	6
8	Wenlong Huang, 2019	Shantou, China	209/165	5
9	Zhang Hong, 2012	Ningxia, China	107/107	5

## Data Availability

The simulation experiment data used to support the findings of this study are available from the corresponding author upon request.
